RETRACTED

# Optimization of trypsin extraction technology of Allium cepa L. polysaccharide by response surface methodology and the antitumor effects through immunomodulation

**DOI:** 10.1080/21655979.2020.1870320

**Published:** 2021-01-20

**Authors:** Yu-Bin Ji, Fu-Ling Wang

**Affiliations:** School of Pharmacy, Engineering Research Center for Medicine, Harbin University of Commerce, Harbin, Heilongjiang, P.R. China; Engineering Research Center of Natural Anticancer Drugs, Ministry of Education, Harbin, Heilongjiang P.R. China

**Keywords:** Polysaccharides of *Allium cepa* L., trypsin-assisted extraction, box-Behnken design, anti-tumor activity, immunomodulation

## Abstract

The trypsin-assisted extraction of polysaccharides from *Allium cepa* L. was optimized using the response surface methodology (RSM). The optimum extraction conditions were extraction temperature, extraction time, extraction pH, and enzyme amount of 37.16°C, 180 min, 8.57, and 5.16%, respectively. Under the optimized conditions, the yield of *A. cepa* L. polysaccharides (ACP) reached 9.69%, which was comparable with the predicted yield (9.73%). Mid- and high-dose ACP significantly inhibited the tumor growth (43.93%) and the tumor inhibition percentage (38.05%), which were more than 30%. The ACP could extend the survival time of H_22_ ascites tumor-bearing mice. Furthermore, the ACP could reduce the thymus and the spleen atrophy and significantly promoted the Con A-induced proliferation of splenocytes and elevated the serum IFN-γ and IL-2 levels. Therefore, the ACP could inhibit the tumor growth in tumor-bearing mice and regulated the immune function of mice.

**Practical Applications**The trypsin-assisted extraction has high efficiency, is carried out through the polysaccharide extraction and the deproteinization at the same time, and is more convenient and fast than traditional methods. No detailed study on the optimization of the trypsin extraction of onion polysaccharides is available. Thus, this experiment aims to use the BBD (4 factors and 3 levels) to optimize the roles of extraction temperature, extraction time, extraction pH, and amount of enzyme on the yield of polysaccharides obtained from the fruit of *A. cepa* L. In addition, when looking for high-quality biological functional principles for the pharmaceutical industry, the antitumor activity of ACP was evaluated. *A. cepa* L. is one of the most widely cultivated and consumed crops worldwide. Polysaccharides are the main active ingredient, and studies have shown that a high intake of *Allium* vegetables is associated with reduced risk of cancers.

## Introduction

*Allium cepa* L. is the most widely cultivated and consumed crop worldwide, represents an important source of dietary phytochemicals with proven antitumor properties [1,2], and is applied in healthcare food. Onion has many biological activities, such as anti-aging, antithrombotic, antitumor, hypolipidemic, and hypoglycemic properties [3]. Plant polysaccharides can fight tumors by inducing the tumor cell apoptosis and improving the immune system [4–7].

RETRACTED

Extraction methods include hot-water, microwave, ultrasound, and enzyme-assisted extraction methods. The extracted polysaccharide contains many proteins. Therefore, the enzyme-assisted extraction method is used [8]. The trypsin-assisted extraction has high efficiency, is carried out through the polysaccharide extraction and the deproteinization at the same time, and more convenient and fast than traditional methods.

The response surface methodology (RSM) can be used as an effective, accurate, and simple tool for the evaluation of multiple parameters and their interactions [9]. Statistical and mathematical techniques may effectively overcome the shortcomings of classic approaches [10,11]. The Box–Behnken design (BBD) is an RSM that is more effective than other methods and can be used to easily arrange and interpret results [12]. The BBD is commonly used to optimize extraction process variables, such as anthocyanins, polysaccharides, and phenolic compounds [13]. The optimal experimental parameters are validated using real samples. The Central Composite Design (CCD) is suitable for multifactor and multilevel experiments with continuous variables. The BBD is suitable for few factors (3 levels and less than 5 factors). The BBD is advantageous because it does not contain any point at the extremes of the cubic region created by the two-level factorial combinations that are prohibitively expensive or impossible to test because of physical constraints on experimentation.

Malignant tumors usually lead to reducing the immune function and the atrophy of immune organs. The spleen and the thymus are key immune organs. IL-2 and IFN-γ are produced by spleen lymphocytes. Thus, cytokines can activate and promote the proliferation of immune cells, which can induce the expression and the release of cytokines and further expand the immune response.

No detailed study on the optimization of trypsin extraction of onion polysaccharides is available. Thus, the experiment aims to use the BBD (4 factors and 3 levels) and optimize the roles of extraction temperature, extraction time, extraction pH, and amount of enzyme on the yield of polysaccharides extracted from the fruit of *Allium cepa* L. (ACP). Besides, the antitumor activity of ACP is evaluated when looking for high-quality biological functional principles for the pharmaceutical industry.

RETRACTED

## Materials and Methods

### Reagents

*Allium cepa* L. was purchased from the wholesale fruit and vegetable market in Harbin, China and identified by professor Bo Yang as the *Allium* onion in the lily family Lilium.

CD-1 mice (SCXK [Beijing] 2006–0009, SPF/VAF, body weight [20 ± 2.0 g], males and females) were provided by the Vital River Laboratory Animal Technology Co., Ltd. (Beijing, China). Murine sarcoma S_180_ cells and mouse H_22_ hepatoma cell lines were obtained from the Cancer Research Institute of Heilongjiang Province (China).

### Enzyme-assisted extraction

Glucose (2 mg) was dissolved in 10 mL water, and the glucose solution was used as standard. Glucose solutions (0.0, 0.2, 0.4, 0.6, 0.8, and 1.0 mL) were extracted using a pipette in a test tube and added with 2.0 mL distilled water and 1.0 mL phenol (6%). The solutions were mixed, added with 5.0 mL concentrated sulfuric acid, mixed immediately, placed at ambient temperature for 5 min, heated for 20 min, and cooled down to 25°C. A UV-visible spectrophotometer (DB-20 R, Dynamica, Australia) was used to evaluate the absorbance of each solution at *λ* = 490 nm. The standard curve was drawn using a polysaccharide concentration (μg/mL) as the abscissa and the absorbance value as the ordinate [14].

The fresh purple onion was skinned, sliced to pieces, and dried. The pieces were ground to obtain a powder, which was sieved at 40 mesh. A certain amount of onion powder was extracted with 80% ethanol (*v:v *= 1:1) for 1.5 h to remove lipids, and the residue was filtered and dried at 60°C. After filtration, the sediment was dried. Pretreated powder was extracted with trypsin solution at a given concentration. The dried onion powder was added with pH buffer and trypsin, subjected to enzymolysis reaction, and stirred using a constant-temperature heating magnetic stirrer. The enzyme deactivation was done at 90°C. After centrifugation (LD4-2A, medical centrifuge factory, Beijing, China) to remove residues for 10 min (3000 rpm), the supernatant was obtained. The extract was concentrated to one-third of the initial volume under reduced pressure at 65°C by using a rotary evaporator. Ethanol (95%) was added to precipitate the concentrate to 80% at 4°C overnight. The precipitate was washed thrice by using an appropriate amount of anhydrous ethanol, acetone, and petroleum ether and freeze-dried to constant weight. The insoluble material was the crude ACP [15].

The content of ACP was determined using the phenol–sulfuric acid method, and D-glucose was used to construct a standard curve. The yield (%) of ACP was calculated as follows:

(1) $$The\;yield\;of\;ACP\left(\%\right)=\frac{\begin{array}{c} Weight\;of\;polysaccharide\;\\ extracted\;from\;Allium\;cepaL.\;\left(g\right) \end{array}}{Weight\;of\;dried\;powder\;sample\left(g\right)}\times 100$$

where *X* is the polysaccharide concentration calculated in accordance with the calibrated regression equation (μg/mL).

RETRACTED

### Single-Factor Experiments

Single-factor experiments were used to evaluate the roles of extraction temperature (30°C, 32°C, 34°C, 36°C, and 38°C), extraction time (60, 90, 120, 150, and 180 min), extraction pH (7.8, 8, 8.2, 8.4, and 8.6), and amount of enzyme (2%, 3%, 4%, 5%, and 6%) on the efficiency of extraction. The independent effect of each factor was determined by changing that factor while all other factors were unchanged.

### Optimization Experimental Design

On the basis of the results of the single-factor experiment, 4 factors and 3 levels of extraction temperature (A), extraction time (B), extraction pH (C), and amount of enzyme (D) were selected as variables to conduct 29 runs of the Box–Behnken design (BBD) [16] experiments (Table 1).

**Table 1.** Experimental design matrix with predicted and observed values

Independent Symbol Variables			Level of Factors				
			−1		0		1
*A*/Temperature (°C) *B*/Time (min) *C*/pH *D*/Enzyme (%)			34 120 8.2 4		36 150 8.4 5		38 180 8.6 6
No. of test	*A*	*B*	*C*	*D*		Yield (%)	
						Experimental	Predicted
1	0	−1	0	−1		6.20	6.35
2	−1	0	0	−1		5.56	5.23
3	0	0	1	1		7.85	7.96
4	0	0	0	0		8.68	8.62
5	0	−1	−1	0		6.75	6.54
6	0	−1	1	0		7.96	8.10
7	0	1	1	0		9.21	9.32
8	0	0	−1	1		7.21	7.28
9	0	0	1	−1		7.79	7.70
10	0	0	0	0		8.38	8.62
11	0	0	0	0		8.72	8.62
12	0	1	0	−1		7.03	7.34
13	0	1	0	1		8.74	8.71
14	0	0	0	0		8.75	8.62
15	−1	−1	0	0		6.29	6.34
16	0	−1	0	1		6.92	6.72
17	0	0	0	0		8.56	8.62
18	1	0	1	0		9.07	8.71
19	−1	0	1	0		6.96	7.05
20	1	1	0	0		9.26	9.20
21	−1	1	0	0		7.05	6.95
22	1	0	0	−1		6.72	6.80
23	−1	0	−1	0		5.58	6.05
24	1	0	0	1		7.23	7.47
25	−1	0	0	1		6.47	6.30
26	0	0	−1	−1		5.92	5.80
27	1	0	−1	0		7.11	7.13
28	0	1	−1	0		8.53	8.30
29	1	−1	0	0		6.74	6.83

## Anti-tumor activity assay in vivo

### Model establishment and administration

The weighed mice after inoculation were randomized and divided into five groups (*n* = 10 per group), i.e., normal control (0.9% normal saline); positive control (astragalus polysaccharides, 100 mg/[kg·day]); and low-, mid-, and high-dose ACP (50, 100, and 200 mg/[kg·day]) groups. The phenol–sulfuric acid method (52.27%) was used to determine the polysaccharide content, and the normal control group was treated with the same volume of normal saline. Food and water were provided to mice. The natural circulation was day and night, and the animal room (temperature, 22°C; humidity, 50–60%) was clean and quiet. The experimental protocol was approved by the Institutional Animal Care and Use Committee of Harbin University of Commerce (Harbin, China).

RETRACTED

### In vivo antitumor experiment

S_180_ tumor‑bearing mice were inoculated with ascites for 7 days and had grown well. Ascites were extracted under aseptic conditions and diluted to a cell suspension with a concentration of 1 × 10^7^ cells/mL with normal saline. The tumor cell suspension (0.2 mL) was subcutaneously injected into the right forelimb armpit of each mouse to create a solid tumor model. All operations were proceeded in an iced bath to maintain the vitality of the cancer cell. After inoculation for 24 h, each group was subjected to sterile intraperitoneal administration, and each mouse was given 0.2 mL drug once a day for 10 consecutive days. Twenty-four hours after the last dose, mice were weighed and sacrificed by cervical dislocation, and the tumor was removed and weighed. The tumor inhibition percentage was calculated in accordance with the following formula. The average tumor weight in the negative control group was less than 1 g and regarded as the performance of the undergrowth of tumor.

(2) $$Tumor\;inhibition\;percentage\left(\%\right)=\frac{\begin{array}{c} average\;tumor\;weight\;of\;the\;control\;group-\\ average\;tumor\;weight\;of\;the\;treatment\;group \end{array}}{average\;tum\;orweight\;of\;the\;control\;group}\times 100$$

### The life-prolonging rate of mice

Mice were intraperitoneally transplanted with 0.2 mL H_22_ (1 × 10^7^ cells/mL) ascites tumor. After 24 h of inoculation, the intragastric administration began per group. Each mouse was treated with 0.2 mL drug daily for 10 consecutive days. Then, the survival time of the mice was recorded.

The rate of extension was calculated using the following formula:

(3) $$Prolongation\;of\;life\;rate\left(\%\right)=\frac{\begin{array}{c} averag\;esurvival\;time\;of\;the\;sample\;group-\\ average\;survival\;time\;of\;the\;control\;group \end{array}}{average\;survival\;time\;of\;the\;control\;group}\times 100$$

### Thymus and spleen index

The thymus and the spleen were resected from the mice, washed with PBS, and weighed. The thymus (TI) and the spleen (SI) indices were calculated using the following formula:

(4) $$TI=\;\frac{thymus\;weight(mg)}{body\;weight(g)}\;\times \;100$$

(5) $$SI=\;\frac{spleen\;weight(mg)}{body\;weight(g)}\;\times \;100$$

### Splenocyte proliferation assay

The spleen from the sacrificed mice was quickly cut into small pieces and pressed to obtain a uniform cell suspension under sterile conditions. Spleen cells were lysed with the lysis buffer (0.83% NH_4_Cl, pH 7.4) for 5 min to remove red blood cells, centrifuged (1000 rpm, 5 min), washed thrice with PBS, and resuspended in the RPMI-1640 medium. The trypan blue dye was used to estimate the cell numbers and viability (over 97%). The spleen cell suspension (5 × 10^6^ cells/mL, 100 μL/well) and Con-A (100 μL/well, 5 μg/mL) were added to the 96-well plate. The same volume of RPMI-1640 medium was added to the control group. Samples were incubated for an additional 68 h (37°C, 5% CO_2_). The MTT solution (5 mg/mL, 10 μL) was added to each well and cultured for another 4 h. Supernatants were carefully removed by pipetting, and 150 μL DMSO was added to each well and oscillated for 10 min to dissolve the purple formazan. The values of OD were evaluated at 570 nm by using a microplate reader (BioTek Instruments, Inc., USA).

RETRACTED

### Assay for IL-2 and IFN-γ

The eyeballs of mice were removed, and blood was collected from eyeballs. Blood samples were collected in test tubes, coagulated at 25°C for 30 min, and centrifuged (1000 rpm, 15 min) to obtain the serum. Following the manufacturer’s instructions (R&D systems, USA), IL-2 and IFN-γ in serum (50 μL) were evaluated using the ELISA kit.

### Statistical Analysis

The Design-expert (version 8.0.7.1) software was used to analyze the experimental design and data and draw the response surface diagram. One-way analysis of variance (ANOVA) was used for pairwise comparisons among groups. p < 0.05 was considered to indicate statistical significance. All measurements were repeated thrice.

## Results and discussion

### Standard Curve

*y* = 0.0281*x* − 0.0023 was the linear regression equation of the glucose standard curve (*R*^2^ = 0.9992), indicating good fitting equation (linearity range: 0–25 μg/mL).

### Single-Factor Experiments

#### Effect of extraction temperature on the ACP YIeld

The highest extraction temperature used was 36°C. The extraction temperature was increased from 30°C to 36°C, and the yield increased. At 36–38°C, the extraction rate decreased. Thus, the temperature range of 34–38°C was adopted for the extraction. One possible reason was that the enzyme activity was remarkably affected by the temperature. At extremely low or high extraction temperature, the enzyme activity may be decreased [17].

#### Effect of extraction time on the ACP yield

As the extraction time increased from 30 min to 150 min, the yield gradually increased until the highest point was reached at 150 min, indicating that the polysaccharide was completely extracted as time passed. After the extraction time reached 180 min, the yield began to decline slightly. The extraction time was 120–180 min. This phenomenon could be attributed to the hydrolysis of polysaccharides during the long extraction process [18].

RETRACTED

#### Effect of pH on the ACP yield

When the pH increased from 7.8 to 8.4, the extraction rate increased and reached the peak value at pH 8.4 and declined at pH 8.6. The extraction pH was 8.2–8.6.

#### Effect of the amount of enzyme on the ACP yield

The 5% amount of enzyme led to the highest extraction yield. Increasing the amount of enzyme resulted in the steady ease of yield. The amount of enzyme of 3–5% was adopted for the extraction.

### Optimization by RSM

Following the data of the single-factor experiment, the roles of extraction temperature (A), extraction time (B), extraction pH (C), and amount of enzyme (D) on the extraction efficiency were determined using the RSM (Figure 1). A second-order polynomial model was established to correlate response variables. The equation was as follows:

**Figure 1.** Role of extraction temperature, extraction time, pH, and amount of enzyme on the yield of *Allium cepa* L. polysaccharide: (a) extraction time, 150 min; pH, 8.4; amount of enzyme, 5%; (b) extraction temperature, 36°C; pH, 8.4; amount of enzyme, 5%; (c) extraction temperature, 36°C; extraction time, 150 min; amount of enzyme, 5%; and (d) extraction temperature, 36°C; extraction time, 150 min; pH, 8.4

*Y* = 8.62 + 0.68A + 0.75B + 0.65 C + 0.43D + 0.44AB + 0.15AC − 0.1AD − 0.13BC + 0.25BD − 0.31 CD − 1.06A^2^ − 0.23B^2^ − 0.32C^2^ − 1.11D^2^.

The result analysis and the coefficient significance test of the quadratic regression equation are shown in Table 2. The model adaptability was evaluated through the lack of fitting test (p > 0.05). Therefore, the regression equation could describe well the true relationship between response values and various factors and determine the optimum extraction conditions through the regression equation.

**Table 2.** Analysis of variance for the quadratic equations of the yield

Source	Sum of Squares	df	Mean Square	*F* Value	*p*-value Prob>F	
Model	34.11	14	2.44	33.97	<0.0001	significant
*A*	5.63	1	5.63	78.50	<0.0001	
*B*	6.69	1	6.69	93.27	<0.0001	
*C*	4.99	1	4.99	69.60	<0.0001	
*D*	2.25	1	2.25	31.42	<0.0001	
*AB*	0.77	1	0.77	10.80	0.0054	
*AC*	0.084	1	0.084	1.17	0.2972	
*AD*	0.040	1	0.040	0.56	0.4676	
*BC*	0.070	1	0.070	0.98	0.3392	
*BD*	0.25	1	0.25	3.42	0.0858	
*CD*	0.38	1	0.38	5.27	0.0376	
*A*^2^	7.29	1	7.29	101.66	<0.0001	
*B*^2^	0.34	1	0.34	4.79	0.0460	
*C*^2^	0.68	1	0.68	9.42	0.0083	
*D*^2^	8.00	1	8.00	111.47	<0.0001	
Residual	1.00	14	0.072			
Lack of Fit	0.91	10	0.091	3.98	0.0976	not significant
Pure Error	0.092	4	0.023			
Cor Total	35.11	28				
*R*^2^	0.9714					
Adj *R*^2^	0.9428					

The model *F* value of 33.97 (p < 0.0001) indicated that the response surface regression model was evident. The possibility of such a large ‘model *F* value’ was only 0.01% due to noise.

RETRACTED

A ‘Prob > F’ value less than 0.0500 or 0.0100 indicated that the model item was valid. A value higher than 0.1000 exhibited that the model item was not evident. In this model, A, B, C, D, AB, A^2^, C^2^, and D^2^ significantly affected the response value (p < 0.01), and the influences of CD and B^2^ on response values were evident (p < 0.05). The rest of the items were all not evident. AC, AD, BC, and BD were not evident effects for the model (Table 2). After excluding their regression coefficients, a prediction model could be given to explain the new situation:

*Y* = 8.62 + 0.68A + 0.75B + 0.65 C + 0.43D + 0.44AB – 0.31 CD −1.06A^2^ – 0.23B^2 –^ 0.32C^2^ – 1.11D^2^.

As shown in Figure 2, the evident order was: extraction time (min) > extraction temperature (°C) > pH > amount of enzyme (%). The Design Expert 8.0.7.1 software revealed that the theoretical optimal conditions for the extraction of ACP were 37.16°C, 180 min, pH 8.57, and 5.16% enzyme.

**Figure 2.** Response surface plots (3-D) and contour plots (2-D) of extraction temperature, extraction time, extraction pH, and amount of enzyme on the yield of ACP

*A* = (*a*-36)/2, *B* = (*b*-150)/30, *C* = (*c*-8.4)/0.2, *D* = (*d*-5)/1, *X*(coded value), *x*(truth value).

The ANOVA was used to assess the significance of each factor and interaction term (Table 2). The *R*^2^ (0.9714), Adj *R*^2^ (0.9428), and Pred *R*^2^ (0.8462) revealed a good relationship between the fitted model and the actual data and the high potential of the model to predict the response. Also, the coefficient of variation was 3.58.

The three-dimensional response surface and contour plots could reflect the strength of the interaction.

### Verification of the model

A potential source of polysaccharides, *A. cepa L*., was used as research material in this study. In recent years, the enzyme-assisted extraction is widely used to extract active ingredients in natural plants. An experiment was conducted to confirm whether the developed extraction model had the best treatment conditions. All experiments were repeated thrice. The optimized conditions (i.e., extraction temperature of 37.16°C, extraction time of 180 min, extraction pH of 8.57, and the amount of enzyme of 5.16%) yielded 9.69% ± 0.06% ACP (*n* = 3), which agreed with the predicted value (9.73%). Compared with the traditional hot-water extraction method, the polysaccharide yield increased by 5.2 percentage points. Results exhibited that the extraction process was stable and reliable, and the extraction rate was high. A high content of polysaccharides could be obtained in accordance with optimal conditions, which was conducive to the study of pharmacological activity and could explain the drug–effect relationship by optimizing the enzymatic extraction process of ACP. The photograph of the ACP powder was taken under a light microscope by using a digital camera (Figure 3 and 4).

RETRACTED

**Figure 3.** Photograph of the ACP powder taken under light microscope (a, 200× magnification) by using a digital camera (b)

**Figure 4.** Effect of ACP on the thymus and the spleen indices of mice with tumor S_180._

### Tumor growth inhibition

Table 3 displays the results of the tumor inhibition percentage. The ACP (different dose groups) significantly inhibited solid S_180_ tumors. The inhibition rates were 24.77%, 43.93%, and 38.05%. Compared with the negative control group, the dose groups were significantly different (p < 0.01).

**Table 3.** Inhibitory effect of the ACP on the solid S_180_ tumor in mice

Group	Dose (mg/(kg·d))	Tumor weight (g)	Tumor inhibition percentage (%)
Control	–	1.0572 ±0.0789	–
APS	100	0.4738 ±0.0331**	55.18
ACP-Low	50	0.7953 ±0.0428**	24.77
ACP-Mid	100	0.5928 ±0.0367**	43.93
ACP-High	200	0.6549 ±0.0551**	38.05

Compared with control group, **p <0.01. Date were expressed as means ± SD (*n* = 10).

### Survival time of mice

All ACP groups prolonged the survival time of H_22_-bearing mice. The survival time of the ACP group was prolonged in a dose-dependent manner (Table 4). The survival times of the high-dose ACP and the control groups were statistically significant (p < 0.01).

**Table 4.** Influence of the ACP on the survival time of mice with tumor H_22._

Group	Dose (mg/(kg·d))	Survival time (d)	Lifeprolong rate (%)
Control	–	10.67 ±1.528	–
APS	100	17.67 ±2.082**	65.60
ACP-Low	50	13.33 ±1.155	24.93
ACP-Mid	100	14.00 ±1.732	31.21
ACP-High	200	16.00 ±2.646**	49.95

Compared with control group, **p <0.01. Date were expressed as means ± SD (*n* = 10).

### Thymus and spleen index

The immune organ index is a preliminary and routine observation index to evaluate the immune function of the body. The thymus, a primary lymphoid organ, is a central immune organ where immune cells are produced, developed, differentiated, and mature. The main function of the thymus is to produce T lymphocytes and participate in cellular immunity. The spleen, a secondary lymphoid organ and the largest peripheral immune organ, is the place where mature lymphocytes settle and produce an immune response, which is related to cellular and humoral immunity. Tumor cells atrophy the thymus and spleen and other important immune organs by inducing lymphocyte apoptosis and reducing the body’s immunity. When the body’s immune status is good, slow tumor development, spontaneous regression, and good prognosis are observed. When the body’s immune function is enhanced, the weight of the immune organs increases. The immune organ index, which can reduce individual differences and objectively reflect the weight change of immune organs, is widely used to evaluate the body’s overall immune level. The TI and the SI of the APS and the ACP groups were markedly higher than those of the control group. The ACP could improve the immune function of tumor-bearing mice.

RETRACTED

### Splenocyte proliferation

The proliferation response of lymphocytes is an important indicator reflecting the activation and the function of lymphocytes. T lymphocytes play the role of the central hub in the body’s immune regulation. By identifying foreign antigens, T lymphocytes proliferate and differentiate into effector cells to mediate the cellular immunity. The strength of its proliferation ability under the stimulation of antigen or mitogen can directly reflect the immune status of the body. When cultured in vitro, the stimulation by mitogens (such as Con A) leads to increased cell volume, vigorous metabolism, and increased protein and nucleic acid syntheses, that is, transformation and proliferation of lymphoblasts. Therefore, the proliferation ability of lymphocytes stimulated by Con A can reflect the influence of drug-mediated immune response. Compared with the control group, the ACP markedly promoted the proliferation of splenocytes stimulated by Con A in S_180_-bearing mice (Figure 5).

**Figure 5.** Effect of the ACP on the spleen lymphocyte proliferation as induced by Con A

### IL-2 and IFN-γ level in S_180_ tumor-bearing mice

Polysaccharides may show their indirect anticancer role via the regulation of immune-related factors, such as IL-2 and IFN-γ levels, and the improvement of the immune response. Data exhibited that ACP could evidently detect IL-2 and IFN-γ levels.

The IL-2 is an important cytokine that regulates the cell-mediated immunity and is produced by activated Th1 cells. The IL-2 produced acts on T cells; induces self-proliferation, differentiation, and function; amplifies immune effects; promotes T cells (Figure 6); and secretes cytokines, such as IFN-γ. The IFN-γ has a strong inhibitory effect on the tumor cell proliferation and the immune regulation. The IL-2 and the IFN-γ positively regulate the functions of macrophages and T cells.

**Figure 6.** Effect of ACP on serum IL-2 and IFN-γ levels

### Conclusion

Onion polysaccharides have antitumor properties and improve immune function. Onion polysaccharides can directly inhibit the growth of tumor tissues in the body, act on multiple links of the immune system, significantly improve the body’s immune function, and reverse the immune suppression state caused by tumor growth. In conclusion, onions have potential use in the therapeutic immunomodulation because they are derived from safe dietary sources and are widely consumed since ancient times. However, the structural properties and the underlying antitumor mechanisms require further study.

RETRACTED

## Highlights

1. The optimum enzymatic extraction process of *Allium cepa* L. polysaccharide was obtained.
2. ACP can inhibit the tumor growth and prolong the survival time of mice.
3. The antitumor activity of ACP may be related to enhancing immune function.
